The article "A stepwise-targeting strategy for the treatment of cerebral ischemic stroke" was retracted in 2022. Reasons: duplicated images; signs of a paper mill; original data or images not available; unreliable data.

# A stepwise-targeting strategy for the treatment of cerebral ischemic stroke

**DOI:** 10.1186/s12951-021-01118-6

**Published:** 2021-11-17

**Authors:** Jingbo Hu, Xueying Tan, Dongwei Wang, Yixuan Li, Hongze Liang, Jiejun Peng, Fengyan Li, Quan Zhou, Peiwu Geng, Shuanghu Wang, Yue Yu, Jin Liu

**Affiliations:** 1 Faculty of Materials Science and Chemical Engineering, Ningbo University, Ningbo, 315211 China; 2 College of Pharmacy, Zhejiang Pharmaceutical College, Ningbo, 315100 China; 3 State Key Laboratory for Managing Biotic and Chemical Threats To the Quality and Safety of Agroproducts, Institute of Plant Virology, Ningbo University, Ningbo, 315211 Zhejiang China; 4 Department of Neurosurgery, The People’s Hospital of Lishui, The Sixth Affiliated Hospital of Wenzhou Medical University, Lishui, 323000 China; 5 Department of Pharmacy, Ningbo Women and Children’s Hospital, Ningbo, 315012 China

**Keywords:** Cerebral ischemic stroke, Stepwise-targeting delivery, Oxidative stress, Melatonin, Micelles

## Abstract

**Background:**

Effective amelioration of neuronal damages in the case of cerebral ischemic stroke (CIS) is essential for the protection of brain tissues and their functional recovery. However, most drugs can not penetrate the blood–brain barrier (BBB), resulting in the poor therapeutic outcomes.

**Results:**

In this study, the derivatization and dual targeted delivery technologies were used to actively transport antioxidant melatonin (MLT) into the mitochondria of oxidative stress-damaged cells in brain tissues. A mitochondrial targeting molecule triphenylphosphine (TPP) was conjugated to melatonin (TPP-MLT) to increase the distribution of melatonin in intracellular mitochondria with the push of mitochondrial transmembrane potential. Then, TPP-MLT was encapsulated in dual targeted micelles mediated by TGN peptide (TGNYKALHPHNG) with high affinity for BBB and SHp peptide (CLEVSRKNG) for the glutamate receptor of oxidative stress-damaged neural cells.TGN/SHp/TPP-MLT micelles could effectively scavenge the overproduced ROS to protect neuronal cells from oxidative stress injury during CIS occurrence, as reflected by the improved infarct volume and neurological deficit in CIS model animals.

**Conclusions:**

These promising results showed this stepwise-targeting drug-loaded micelles potentially represent a significant advancement in the precise treatment of CIS.

**Graphical Abstract:**

**Supplementary Information:**

The online version contains supplementary material available at 10.1186/s12951-021-01118-6.

## Introduction

Cerebral ischemic stroke (CIS) is characterized by its high morbidity, high mortality, high disability and high recurrence rate, thus it seriously endangers human health [1]. In the case of CIS, the natural recanalization of the arteries in the brain tissue of patients who have not received thrombolytic treatment may cause over-reperfusion, while the recanalization of the blood vessels of patients treated with thrombolytic therapy may realize partial effective reperfusion [2, 3]. However, due to damage to the structural and functional integrity of the microvasculature of the brain tissue, reperfusion damage may be caused as a result of the neurological injury cascade triggered by disruption of the blood–brain barrier and auto-regulatory failure [4, 5]. Therefore, effective amelioration of neuronal damage in the case of CIS is essential for the protection of brain tissues and their functional recovery.

At present, there are many varieties of clinical antioxidants, such as acetylcysteine and melatonin, while the overall therapeutic outcomes are often unsatisfactory, which is mainly due to: (i) The existence of the blood–brain barrier (BBB) which has a tight structure composed of brain capillary endothelial cells, astrocyte terminal feet, adventitial cells and vascular basement membranes, leads to the situation that there is almost no cellular gap between cells but an efficient efflux system (such as P-glycoprotein) on BBB. Therefore, this tight BBB makes it difficult for 98% of small molecule drugs and almost all macromolecular drugs to enter the nerve cell [6, 7]. (ii) The drugs show a whole-brain distribution after entering the brain tissue and cannot be concentrated on the lesion. Considering the extreme sensitivity of nerve cells to injury, the whole-brain distribution of drugs not only reduces the concentration of drugs reaching the site of injury, thus weakening the therapeutic effect, and may also induce serious toxic side effects on the normal central nerve. Hence, the key to CIS antioxidant therapy is how to enable as many antioxidants as possible to cross the BBB, achieve active targeted delivery of oxidative stress-damaged nerve cells and intracellular mitochondria.

Melatonin, as an indole hormone secreted by the pineal gland, has many important biological functions, such as anti-inflammatory, antioxidant, anti-tumor functions and free radical scavenging in the body [8, 9]. Melatonin could protect nerve cells against lipopolysaccharide-induced oxidative stress damage, acute neuroinflammation, and apoptotic neurodegeneration [10]. However, melatonin is limited by its short half-life and easy to be metabolized in the body, as well as lack of selective specificity for nerve cells in brain tissues, thus its efficacy is often unsatisfactory. Therefore, it is necessary to improve the therapeutic effect of melatonin in CIS with the help of drug delivery systems alter the distribution of the drug in the body.

The ability to specifically transport drugs to the pathological lesion of brain tissues of great importance for the treatment of CIS. Currently, there are two main approaches to facilitate drug passage through BBB for the treatment of CIS: (1) Nasal administration, after which, BBB can bypass the olfactory and trigeminal nerve pathways for direct transport into the brain [11, 12], the way of which is convenient but still brings many problems, such as the low amount of polar macromolecular drugs into the brain (only 0.01% ~ 0.1% of the administered dose), easily affected absorption by pathological conditions such as cold and rhinitis as well as individual differences [13]; (2) Nanoparticle drug delivery systems for drug delivery, i.e., taking advantage of a variety of allosteric receptors and transporters on brain capillary endothelial cells, select their corresponding ligands as the target functional base, modify the surface of the drug delivery system, and mediate its trans-BBB transport into the brain [14, 15]. This strategy can not only effectively overcome the barrier of BBB, but also increase the stability of the drug in the body and prolong its half-life in body system. It is one of the most mature brain-targeting strategies and has received wide attention.

Based on the above background, a mitochondrial targeting molecule triphenylphosphine (TPP) was conjugated to melatonin (TPP-MLT) and increased the distribution of melatonin in intracellular mitochondria with the push of mitochondrial transmembrane potential [16], aiming to effectively scavenge and inhibit intracellular production of ROS under pathological conditions. Secondly, TPP-MLT was encapsulated in two-stage targeted micelles mediated by TGN peptide (TGNYKALHPHNG) with high affinity for BBB and the SHp peptide (CLEVSRKNC) with high affinity for the glutamate receptor of oxidative stress-damaged neural cells with up-regulated specificity during the occurrence of CIS [17, 18]. TGN/SHp/TPP-MLT micelles increase the targeted transport of TPP-MLT to brain tissues, and further act on damaged cells by the mediation of SHp peptide to enhance the drug therapeutic effect, thus effectively protecting neural cells, and achieving the precise treatment of CIS.

## Materials and methods

### Materials

TGN peptide and SHp peptide were purchased from ChinaPeptides (Shanghai, China). Melatonin and (4-Carboxybutyl)triphenylphosphonium bromide were purchased from Aladdin Bio-chem Technology (Shanghai, China). Maleimide-poly(ethylene glycol)2000-poly (lactic acid)5000 (Mal-PEG-PLGA) and methoxy poly (ethylene glycol)2000-poly(lactic acid)5000 (MePEG-PLGA) were purchased from Xi’an ruixi Biological Technology (Xi’an, China). JC-1 and DCFH-DA were purchased from Invitrogen (Carlsbad, USA). MTT was purchased from Solarbio technology (Beijing, China). Fetal bovine serum (FBS), DMEM media, PBS buffer, trypsin/EDTA, and penicillin–streptomycin were purchased from Hyclone Laboratories (Logan, USA). Superoxide dismutase (SOD) and Malonaldehyde (MDA) were purchased from Nanjing jiancheng Bioengineering Institute (Nanjing, China).

### Synthesis and characterization of TPP-MLT

TPP-MLT was synthesized as shown in Fig. 1A. To a solution of (4-carboxybutyl)triphenylphosphonium bromide 1 (1.33 g, 3 mmol) in dry dichloromethane (20 mL) was added thionyl chloride (1.5 mL). The reaction mixture was heated to 90℃ and refluxed for 3 h until no starting material of 1 was exist. The resulting mixture was cooled to room temperature and concentrated to dry. The white solid of 2 was obtained and used in the following step without further purification.

**Fig. 1:** Melatonin derivative TPP-MLT and its antioxidant activity. **A** Synthetic route of TPP-MLT (compound 3). **B** ^1^H NMR spectrum of TPP-MLT (500 MHz, Chloroform-d). **C** Mass spectrum of TPP-MLT. **D** The MLT content in mitochondria of PC-12 cells treated with MLT and TPP-MLT (n = 6, **P < 0.01, *P < 0.05). **E** Expression levels of ROS in PC-12 cells treated with MLT and TPP-MLT. DCFH-DA fluorescent probes as ROS indicator. Scale bar, 50 μm. **F** The changes of mitochondrial membrane potential in PC-12 cells treated with MLT and TPP-MLT. Scale bar, 50 μm. **G** Cell viability of PC-12 cells treated with MLT and TPP-MLT (n = 6, *P < 0.05). **H** PC-12 cells were stained with calcein AM (green) and EthD-1 (red) to visualize live and dead cells. Scale bar, 200 μm

In a round-bottom flask was added melatonine (0.93 g, 4 mmol), triethylamine (0.56 mL, 4 mmol) and dry dichloromethane (20 mL). Then a solution of compound 2 produced above in dry dichloromethane (10 mL) was added dropwise into the mixture under ice bath. After addition, the reaction mixture was stirred at room temperature over 16 h. Then the mixture was concentrated to dry and the crude product was purified by column chromatography using MeOH/DCM (v/v = 1/10) as eluent to get 1.42 g white solid 3, yield 72%.

### Mitochondrial distribution of TPP-MLT

The mitochondrial distribution of TPP-MLT in PC-12 cells (rat adrenal pheochromocytoma cell line) was determined quantitatively, free MLT as control. PC-12 cells were seeded in 6-well plates at a density of 1 × 10^5^/mL, and incubated with various concentrations of MLT and TPP-MLT (MLT, 2, 4, 8, 16 and 32 μg/mL). After 2.0 h, cells were collected by centrifugation (1000 rpm, 5 min) and washed twice by PBS, and mitochondria were collected using a mitochondrion isolation kit (Sigma-Aldrich, USA). The drug was dissolved with DMSO and determined by UPLC-MS/MS (Acquity I-Class UPLC and a XEVO TQD triple quadrupole mass spectrometer, Waters Corp.).

### Synthesis and characterization of TGN-PEG-PLGA and SHp-PEG-PLGA

TGN-PEG-PLGA was synthesized via maleimide-thiol coupling reaction between TGN and Mal-PEG-PLGA at a 1:1 molar ratio under the protection of nitrogen for 4 h. After reaction, the crude product was purified by dialysis(MWCO: 3.5 kDa) against deionized water for 48 h, followed by lyophilization. SHp-PEG-PLGA was prepared in the same way. The proton spectra of TGN-PEG-PLGA and SHp-PEG-PLGA were confirmed using NMR spectrometer (Bruker, 500 Hz), DMSO-*d*_*6*_ as solvent.

### Preparation and characterization ofTGN/SHp/TPP-MLT micelles

TGN/SHp/TPP-MLT micelles with a 1:1 ratio of TGN and SHp were constructed by solvent diffusion, and the hydrophobic TPP-MLT was encapsulated in the hydrophobic core of the micelles. SHp-PEG-PLGA, TGN-PEG-PLGA and MePEG-PLGA at a molar ratio of 1:1:3 were dissolved in 0.5 mL ethanol, and then mixed with another 0.5 mL ethanol with TPP-MLT. The mixed solution was added into 10 mL of deionized water and stirred for 10 min at room temperature, and then transferred to a dialysis bag (MWCO: 3.5 kDa) and dialyzed with deionized water to remove ethanol. The resulting dialysate was centrifuged at 5000 rpm for 10 min, and the insolubilized TPP-MLT was removed to obtain TGN/SHp/TPP-MLT micelles.

10 mg TGN/SHp/TPP-MLT micelles were dispersed in 10 mL deionized water, and the zeta potential and particle size of TGN/SHp/TPP-MLT micelles were determined by dynamic light scattering (Malvern, Zetasizer 3000HS).

0.1 mg/mL TGN/SHp/TPP-MLT micelles were instilled on the 300-eye copper mesh, then air-dried and negatively dyed by 1% uranyl acetate solution for 1 min to remove the redundant staining solution, and the morphological structure was observed under the transmission electron microscopy (Hitachi, H7650).

The in vitro release behavior of TGN/SHp/TPP-MLT micelles was investigated by the dialysis method [19]. The weighted free TPP-MLT, TPP-MLT micelles and TGN/SHp/TPP-MLT micelles (equal TPP-MLT) were transferred into the dialysis bag (MWCO: 3.5 kDa) and loaded into a centrifuge tube containing 40 mL of pH 7.4 PBS. After shaking at 80 rpm under 37 °C, it was sampled by 1 mL at 0.5, 1, 2, 3, 4, 6, 8, 10, 12 and 24 h respectively, and then replenished with release medium of the same volume. The TPP-MLT content in the release medium was quantified by UPLC-MS/MS. In addition, the release behavior of TGN/SHp/TPP-MLT micelles in pH 7.4 PBS containing 10% fetal bovine serum was also assessed as our previous study [20].

### Stability of TGN/SHp/TPP-MLT micelles

The lyophilized TGN/SHp/TPP-MLT micelles were stored at 4 °C for various periods of time, and average diameter, PDI and drug loading were measured. In addition, the in vitro release behavior of TGN/SHp/TPP-MLT micelles after stored at day 7 was also investigated.

### Cytotoxicity

The cytotoxicity of TGN/SHp/TPP-MLT micelles was investigated by MTT using bEnd.3 and PC-12 cells as model cells [21]. Cells were seeded in 96-well cell culture plates at a density of 1 × 10^3^per well. After the cells adhered overnight, TGN/SHp/TPP-MLT micelles with a series of concentrations were added, with cells added with PBS solution of the same volume as a comparison. After incubation for 24 h, 10 µL of MTT solution was added to each well for further incubation for 4 h. Then the supernatant was discarded, 100µL of DMSO was added to dissolve the purple precipitate formazan, and the absorbency was measured at 570 nm to calculate the survival rates.

Cell viability of PC-12 cells was further visualized by the LIVE/DEAD Viability/Cytotoxicity Kit (Invitrogen, USA) [22]. Cells were seeded in 12-well cell culture plates at a density of 1 × 10^3^per well, and incubated overnight.H_2_O_2_ solution (200 µM, 2 h) was added to induce oxidative stress damage of PC-12 cells, and free TPP-MLT and TGN/SHp/TPP-MLT micelles (TPP-MLT, 10 μM) were added respectively for further incubation. Then, cells were washed with cold PBS, and then stained with calcein-AM (green) and EthD-1 (red)according to the manufacturer's protocol, followed by observation under an inversed fluorescent microscope (Zeiss, Axio Observer 5).

### Hemolysis test

20 mL of rabbit blood was added in a glass tube and stirred by glass rod to remove fibrous proteins. Normal saline of quintuple volume was added before shaking up and centrifugation at 1500 rpm for 15 min. Then the supernatant was discarded and the precipitated erythrocytes were washed 2 more times as described above until the supernatant did not appear red, and the obtained erythrocytes were made into a 2% suspension by normal saline for later use. The hemolysis test was divided into 7 groups which are the deionized water group, normal saline group as well as the TGN/SHp/TPP-MLT micelle groups of 10, 20, 40 and 80 µg/mL. Each tube was left stationary at 37 ℃ for 1 h for observation after applying samples with the deionized water group as the positive control and the normal saline group as the negative control to determine the OD value and calculate the hemolysis ratio [23].

### Cellular uptake

To investigate the internalization of TGN/SHp micelles, fluorescent probe cy3 was used to label TGN/SHp micelles, and TGN/SHp/cy3 micelles were prepared using the method for TGN/SHp/TPP-MLT micelles. The bEnd.3 cells (mouse brain microvascular endothelial cells) were seeded in 6-well plates at 2 × 10^5^ cells per well and incubated with TGN/SHp/cy3 micelles for 0.5 h and 2.0 h, respectively. TGN/cy3micelles, SHp/cy3 micelles, cy3 micelles and free cy3 were used as control. After incubation, the cells were washed three times with PBS (pH 7.4), fixed in 4% paraformaldehyde for 30 min, and then observed by an inversed fluorescent microscope. The internalization of TGN/SHp/cy3 micelles by bEnd.3 cells was further analysed by flow cytometry (Beckman Coulter, CytoFlex S).

PC-12 cells were seeded in 6-well plates at 2 × 10^5^ cells per well and incubated overnight. Cells were treated with H_2_O_2_ (200 μM) or PBS for 4 h, and then incubated with TGN/SHp/cy3 micelles for 0.5 h and 2.0 h, respectively. TGN/cy3 micelles, SHp/cy3 micelles, cy3 micelles and free cy3 were used as control. After incubation, intracellular fluorescence signals were observed by an inversed fluorescent microscope. The internalization of TGN/SHp/cy3 micelles by oxidative stress-damaged PC-12 was also analysed by flow cytometry.

### Establishment of blood brain barrier and transmembrane activity

The bEnd.3 cells were seeded at a density of 5 × 10^4^ cells/well on the inserts of Transwell culture plates with a volume of 0.5 mL for the upper layer and 1.5 mL for the lower one. The culture continued for one week with the culture medium changed every two days, and the transepithelial electrical resistance (TEER) of each layer of cells was measured by a transepithelial resistance meter after 7 days [24].

In addition, the compactness of the monolayer cells was evaluated by measuring the transmittance of horseradish peroxidase (T_HRP_) [25]. 500 ng of horseradish peroxidase (HRP) was dissolved in 0.5 mL of serum-free culture medium and placed on the upper layer of the culture plate; 1.1 mL of the culture medium was added to the lower layer, and 0.5 mL of the culture medium was taken from the upper and lower layers of the culture plate at different time points. The T_HRP_ was calculated by adding 100 µL of catalase as the substrate and incubating for 3 min, then adding 50 µL of sulfuric acid (1 M) to abort the reaction and measuring the optical density value at 450 nm.

Monolayer cells with their TEER > 200Ω/cm^2^ can be used for BBB transport test by adding 50 µg/mL of TGN/SHp/cy3 micelles to the upper layer of Transwell inserts, with TGN/cy3 micelles, SHp/cy3 micelles, cy3 micelles and free cy3 as the control, and D-Hanks liquid as the transport medium. The cy3 fluorescence intensity (Ex = 548 nm, Em = 568 nm) was measured by a spectrophotofluorometer by sampling 100 µL at 0.5, 1 and 2 h time points while adding an equal volume of fresh D-Hanks solution, to calculate the transmittance of TGN/SHp/cy3 micelles in monolayers.

### Establishment of CIS animal model

BALB/c mice were used as model animals for establishing an animal model of transient left middle cerebral artery occlusion (MCAO) by thread occlusion [15]. The mice, with the neck de-haired and sterilized, were fixed in the supine position on a small-animal temperature-controlled operating table. The left common carotid artery was isolated after an anterior median carotid incision, then the proximal end of the carotid artery was ligated with sutures, and the common and internal carotid arteries were closed by vascular clips. The cerebral thrombus nylon wire was inserted from the back of an oblique incision on the external carotid artery from the bifurcation of the common carotid artery. The proximal end was ligated by ligature wire and the external carotid artery was cut. Then the vascular clamp of the internal carotid artery was opened, and the nylon wire was rapidly pushed into the internal carotid artery. Resistance was felt when the wire entered at a depth of approximately 20 mm from the bifurcation of the common carotid artery, which indicates that the wire had reached the position of the left middle cerebral artery and you should stop pushing the wire. The wire was removed 1 h after the ligature of external carotid artery which was knotted at the root by a suture, and the vascular clamp of the common carotid artery was opened to allow reperfusion of blood flow into the brain. The mice were maintained at 37 ± 0.5 °C throughout the operation.

### Bio-distribution

To investigate the brain distribution of TGN/SHp micelles in CIS mice, near-infrared fluorescent probe Dir was used to label TGN/SHp micelles, and TGN/SHp/Dir micelles were prepared using the method for TGN/SHp/TPP-MLT micelles. TGN/SHp/Dir micelles (Dir, 20 nmol/kg) were intravenously injected at 2 h after MCAO. After washed by PBS,the brain tissues were dissected for ex vivo fluorescence imaging using the In-Vivo imaging system (Perkin Elmer, IVIS Lumia III).

Then, the distributions of TPP-MLT in various tissues after treated with TGN/SHp/TPP-MLT micelles (TPP-MLT, 5 mg/kg) were quantificationally determined by UPLC-MS/MS, free TPP-MLT and TPP-MLT micelles as control. At 0.5, 2 and 8 h after the administration, the CIS mice were put to death with the heart, liver, spleen, lung, kidney and brain tissues taken for sample introduction and analysis after sample treatment to measure the concentrations of TPP-MLT in various tissues. Tissue samples were taken and rinsed with PBS, then absorbed dry by filter paper after washing by PBS before weighing and grinding in the ice bath with a homogenizer. Then the homogenate was centrifuged at 5,000 rpm for 10 min. 100 µL of supernatant was taken and added with acetonitrile until reaching 1 mL, then whirled for 5 min and centrifuged at 5,000 rpm for 10 min before blowing dry the supernatant with nitrogen. The residue was dissolved with 200µL of acetonitrile and centrifuged, and then the supernatant was taken for analysis.Likewise, the TPP-MLT contents in the ischemic and normal sides of the brain tissues were examined to evaluate the selective distribution ability of TGN/SHp/TPP-MLT micelles to the infarct area of brain tissues.

### ROS detection

Intracellular reactive oxygen species (ROS) production of PC-12 cells was labelled using DCFH-DA fluorescent probes [26]. PC-12 cells were seeded at a density of 1 × 10^4^ per well in 12-well plates and incubated under 5% CO_2_ at 37 °C. After that, H_2_O_2_ solution (200 µM, 2 h) was added to induce oxidative stress damage in PC-12 cells, and free MLT, free TPP-MLT and TGN/SHp/TPP-MLT micelles (TPP-MLT, 10 µM) were added respectively for further incubation for 12 h.The culture medium was then discarded, DCFH-DA was diluted by serum-free culture medium to a final concentration of 10 µM, and probes were loaded to PC-12. The added DCFH-DA should fully cover the cells for incubation for 20 min under 37 °C. Cells were washed with serum-free cell culture medium to remove DCFH-DA fluorescent probes that did not enter the cells, and were observed and photographed under a fluorescent inverted microscope.

### Mitochondrial membrane potential

JC-1 probe (E_x_ = 488 nm, E_m_ = 535 nm) was used to assess the changes in mitochondrial membrane potential (MMP) in oxidative stress-damaged PC-12 cells [27]. Cells were seeded at a density of 1 × 10^4^ per well in 12-well and incubated overnight. Then H_2_O_2_ solution (200 µM, 2 h), and free MLT, free TPP-MLT and TGN/SHp/TPP-MLT micelles (TPP-MLT, 10 µM) were added respectively for further incubation for 12 h. After treatment, culture medium containing JC-1 probe (10 µg/mL) was added and incubated for 15 min. Cells were washed with serum-free cell culture medium to remove JC-1 probe that did not enter the cells, and were observed and photographed under a fluorescent inverted microscope.

### Apoptosis detection

PC-12 cells were seeded at a density of 1 × 10^5^ per well in 6-well and incubated overnight. H_2_O_2_ solution (200 µM, 2 h), and free TPP-MLT and TGN/SHp/TPP-MLT micelles (TPP-MLT, 10 µM) were added respectively for further incubation for 12 h. Then, cells were collected, resuspended with PBS, incubated with annexin V-FITC/propidium iodide [28], and analyzed by flow cytometer (Beckman Coulter, CytoFlex S).

### Western blot

Sample treatment was referred to our previous study [29]. Anti-Cytochrome C (1:5000, Abcam), anti-Cleaved Caspase-3 (1:5000, Abcam) and anti-Cleaved Caspase-9 (1:5000, Abcam) antibodies were used to detect the effects of TGN/SHp/TPP-MLT micelles on the mitochondrial apoptosis pathway. The cytosolic and mitochondrial fractions of PC-12 cells were isolated by standard differential centrifugations using a a mitochondrion isolation kit (Sigma-Aldrich, USA). Normalization was ensured by VDAC-1 and β‐actin, and the target bands were quantified by ImageJ software.

### Neurological deficit score

Sham-operated mice was taken as negative control and MCAO mice were injected with saline, free TPP-MLT and TGN/SHp/TPP-MLT micelles at the TPP-MLT concentration of 5 mg/kg, respectively. Neurological deficit scores were evaluated at 24 h after MCAO and scored according to Longa’s 6-grade and 5-point scale with the following standards: 0 point: No symptom; 1 point, impairment of extending contralateral forelimb during tail suspension; 2 points, injury to the contralateral forelimb flexion during tail suspension; 3 points, slight leaning to the paralyzed side while walking; 4 points, heavy leaning to the paralyzed side while walking; 5 points, unable to walk on its own, impaired consciousness [30].

### Magnetic Resonance Imaging

CIS mice were anesthetized by intraperitoneal injection of sodium pentobarbital (80 mg/kg) and placed in the prone position, and brain tissues were observed with the help of a 3.0 T whole body magnetic resonance imaging system (GE Healthcare, MR750). Each of the 11 layers was set as 2 mm with 0 mm gap.

### 2,3,5-triphenyltetrazolium chloride (TTC) staining

The brain tissue was removed intact after execution, and the brain was evenly cut into six coronal sections with a thickness of 1 mm. The brain slices were immersed in 2% TTC solution, incubated in 37 ℃ water bath for 30 min, then stained and fixed in 4% paraformaldehyde for 24 h for photographing. The area of infarction and the percentage of hemispherical swelling were analyzed by ImageJ software (the red area was normal brain tissues, and the white area was the infarcted area) [31].

### Histological analysis

The isolated brain tissues were fixed in 10% formaldehyde for 24 h, routinely embedded in paraffin and sectioned, then placed at 60 °C for 2 h before dewaxing by xylene and eluting by alcohol gradiently, and at last routinely stained with HE and sealed by resin before observation with an inverted microscope.

### Detection of oxidative stress

An appropriate amount of brain tissues was taken and added with cold normal saline according to the weight-to-volume ratio (the ratio of tissue to normal saline was 1:9), then cut to pieces and centrifuged at 4000 r/min for 10 min to make 10% brain tissue homogenate. The levels of superoxide dismutase (SOD) and malondialdehyde (MDA) were determined according to the kit manual (Nanjing Jiancheng Bioengineering Institute, China).

### Statistical analysis

Data were processed using SPSS 14 statistical software. The measurement data were expressed as mean ± standard error, and statistical differences were tested by one-way ANOVA followed by the analysis using t-test and post hoc Fisher’s test after the homogeneity test of variance. The tested differences were considered statistically significant if *P* < 0.05.

## Results

### Characterization and anti-antioxidant activity of TPP-MLT

The synthetic route of TPP-MLT (compound 3) was illustrated in Fig. 1A was successfully obtained in two steps. TPP-MLT was characterized by NMR spectra and ESI–MS analysis (Fig. 1B and C). ESI–MS, m/z 577.21 ([M—Br]^+^ calcd for C_36_H_38_N_2_O_3_P^+^, 577.26). ^1^H NMR (500 MHz) δ (ppm) 10.67 (s, 1H), 7.98–7.89 (m, 4H), 7.86–7.75 (m, 10H), 7.26–7.21 (m, 1H), 7.13 (d, *J* = 15 Hz, 1H), 7.05 (d, *J* = 15 Hz, 1H), 6.75–6.70 (m, 1H), 3.79 (s, 3H), 3.65–3.61 (m, 2H), 3.38–3.26 (m, 4H), 2.82–2.75 (m, 1H), 2.54 (d, *J* = 15 Hz, 2H), 2.34–2.27 (m, 1H), 1.84 (s, 3H), 1.80–1.68 (m, 1H), 1.63–1.56 (m, 1H).

The mitochondrial distribution of TPP-MLT in PC-12 cells was determined quantitatively by UPLC-MS/MS, free MLT as control. As shown in Fig. 1D, the distribution of MLT in mitochondria in TPP-MLT group was significantly higher than that in MLT group, demonstrating that the mitochondrial targeting molecule TPP modification significantly increased the directional distribution of MLT in mitochondria (**P < 0.01, *P < 0.05). DCFH-DA itself has no fluorescence and can be hydrolyzed into DCFH by esterase upon entry into the cell, while DCFH cannot permeate the cell membrane, thus allowing successful loading of the probe into cells [32]. Intracellular ROS can oxidize non-fluorescent DCFH to generate fluorescent DCF so as to reflect the level of intracellular ROS production. As shown in Fig. 1E, normal cells have little fluorescence, while hydrogen peroxide induces oxidative stress-damaged cells to produce large amounts of ROS, which exhibits strong green fluorescent signals. The intracellular ROS levels were reduced differentially after MLT and TPP-MLT treatment, and TPP-MLT was superior to MLT due to the advantage that TPP allowed more MLT to be distributed directionally to mitochondria, the main sites of ROS production.

The decrease in mitochondrial membrane potential, as an early sign of cell apoptosis, is often detected with the aid of the JC-1 fluorescent probe. The JC-1 fluorescent probe was adopted in this study to investigate the effect of TPP-MLT on apoptosis of PC-12 cells. At higher mitochondrial membrane potentials, JC-1 aggregates in the mitochondrial matrix to form a polymer that exhibits red fluorescence. Whereas when the membrane potential is low, JC-1 is unable to aggregate in the matrix with JC-1 of monomeric and showing green fluorescence [33]. The change of mitochondrial membrane potential is indicated by a shift in the color of the fluorescent probe, and the relative ratio of red to green fluorescence is employed to measure the degree of mitochondrial depolarization with the results as shown in Fig. 1F. The induction of H_2_O_2_ made the PC-12 cell membrane potential decrease rapidly, which demonstrated that the red fluorescence signal became weaker and the green signal enhanced, while the mitochondrial membrane potential was improved to different degrees after the intervention of MLT and TPP-MLT, in which the effect of TPP-MLT was better than that of MLT, further demonstrating the advantages of the antioxidant TPP-MLT with mitochondrial targeting performance.

A model of cells injured by oxidative stress was constructed by H_2_O_2_ induction, and the cell survival rate after TPP-MLT intervention was examined by the MTT method. As shown in Fig. 1G, both MLT and TPP-MLT were effective in improving the survival of oxidative stress-damaged cells, with the efficacy of TPP-MLT being significantly better than that of MLT. Calcein AM (green, live cells) and Ethd-1 (red, dead cells) fluorescent probes were further used for investigating the cell survival of PC-12 cells after MLT and TPP-MLT treatment. The results are as shown in Fig. 1H and Additional file 1: Fig. S1. H_2_O_2_ induced oxidative stress damage to cells, which in turn led to massive cell death. MLT and TPP-MLT were effective in improving cell survival, with TPP-MLT significantly better in effect than MLT as well.

### Characterization of TGN/SHp/TPP-MLT micelles

Both TGN-PEG-PLGA and SHp-PEG-PLGA were synthesized via maleimide-thiol coupling reaction, and ^*1*^*H*NMR results were shown in Additional file 1: Fig. S2 and S3. The characteristic peak of the TGN peptide (A1, 7.0–9.0 ppm) was visible in the TGN-PEG-PLGA (A2). Similarly, the characteristic peak of the SHp peptide (B1, 8.0 ppm) was also present in the synthetic product SHp-PEG-PLGA (B2).

Then, TGN/SHp/TPP-MLT micelles were prepared via solvent diffusion. TGN-PEG-PLGA, SHp-PEG-PLGA and MePEG-PLGA with a ratio of 1:1:3 were used as carrier materials to construct drug-loading micelles, and all of these three grafts are amphipathic. TGN-PEG, SHp-PEG and MePEG all act as hydrophilic groups, while PLGA, as a hydrophobic group, can form micelles with unique nucleus-shell structures in aqueous media. The hydrophobic core formed by PLGA can be used for loading TPP-MLT, while the hydrophilic shell allows the micelles to remain stable in aqueous media. TGN/SHp/TPP-MLT micelles were prepared using solvent diffusion (Fig. 2A) by rapidly injecting the mixed ethanol solution of TGN-PEG-PLGA, SHp-PEG-PLGA, MePEG-PLGA and TPP-MLT in different ratios into the aqueous solution, and the amphiphilic materials self-aggregated to form micelles, while the hydrophobic TPP-MLT entered into the hydrophobic core of PLGA due to the increased polarity of the medium. Deionized water dialysis further permeated ethanol out of the dialysis bag, which had a MWCO of 3.5 kDa. The drug-loading micelles would not extravasate out of the bag, but the ethanol with a lower molecular weight continued to extravasate out of the dialysis bag due to the concentration difference. With the dialysis media changed repeatedly, the final ethanol could be eliminated.

**Fig. 2:** Preparation and characterization of TGN/SHp/TPP-MLT micelles. **A** Preparation process diagram of TGN/SHp/TPP-MLT micelles. **B** Transimission electron microscope images and dynamic light scattering of TPP-MLT micelles and TGN/SHp/TPP-MLT micelles. Scale bar, 100 nm. **C** The drug loading of TPP-MLT micelles and TGN/SHp/TPP-MLT micelles after various feeding ratio. **D** In vitro release curves of TGN/SHp/TPP-MLT micelles, free TPP-MLT and TPP-MLT micelles as control. **E** In vitro release curves of TGN/SHp/TPP-MLT micelles in pH7.4 PBS containg 10% fetal bovine serum (FBS). **F**–**H** The changes in diameter, PDI and drug loading of TGN/SHp/TPP-MLT micelles kept in 4 °C at different days, TPP-MLT micelles as control(n = 6). **I** In vitro release curves of TGN/SHp/TPP-MLT micelles after stored at day 7, day 1 as control (n = 6)

The loading of TPP-MLT into the TGN/SHp micelles did not induce significant changes in the particle sizes and zeta potential of these micelles (Additional file 1: Table S1). With the increase of TPP-MLT feeding ratio, no significant enhanced drug loading was observed when feeding ratio ≥ 10%. The micellar size change tendency was similar to that of TPP-MLT load increase. The particle size of TGN/SHp/TPP-MLT micelles was 97.5 ± 4.9 nm when the dosing of TPP-MLT was 10%. The particle size of blank TGN/SHp micelles was slightly more than TGN/SHp/TPP-MLT micelles with 5% feeding ratio of TPP-MLT (88.6 ± 5.3 *vs.* 84.2 ± 4.8), which was associated with hydrophobic interaction between the hydrophobic PLGA and the encapsulated TPP-MLT. After reaching a certain loading capacity, with the increase of TPP-MLT content, the particle size of the micelles gradually increased. The transmission electron microscope was adopted to observe the morphology of TGN/SHp/TPP-MLT micelles, and micelles with 10% of the dose were selected for observation. As shown in Fig. 2B, the micellar morphology was spherical with uniform particle size.

The content of TPP-MLT in TGN/SHp/TPP-MLT micelles was determined by organic solvent extraction. The TGN/SHp/TPP-MLT micelles were dissolved in DMSO and PEG-PLGA could not aggregate in the organic phase to form micelles. Therefore the concentration of TPP-MLT could be determined after dilution by the mobile phase, and then the drug loading capacity of TGN/SHp/TPP-MLT micelles could be further determined with the results as shown in Fig. 2C. The content of TPP-MLT in TGN/SHp/TPP-MLT micelles increased from 4.29 ± 0.55% to 8.94 ± 0.89% when the dose was increased from 5 to 10%, while the increase was not significant with further increase in the dose. Therefore, TGN/SHp/TPP-MLT micelles with a dose of 10% were used for the follow-up experiment.

The in vitro drug release behavior of TGN/SHp/TPP-MLT micelles was investigated by the dialysis bag method, with free TPP-MLT and TPP-MLT micelles as the control. The results are shown in Fig. 2D, the release of free TPP-MLT was complete around 12 h while the release of TPP-MLT could be maintained for 24 h after encapsulated in micelles, and the modification of TGN peptide and SHp peptide had no effect on the release of TPP-MLT. In addition, pH 7.4 PBS containing 5% fetal calf serum (FBS) was used as the release medium to investigate the release behavior of TGN/SHp/TPP-MLT micelles in this medium, with the results as shown in Fig. 2E. The presence of 5% FBS had no effect on the release behavior of TGN/SHp/TPP-MLT micelles.

The in vitro stability of TGN/SHp/TPP-MLT micelles was investigated via monitoring particle size, PDI, drug loading and drug release behavior at pre-designed times. As shown in Fig. 2F–I, no significant changes were observed in particle size, PDI, drug loading and drug release behavior of TGN/SHp/TPP-MLT micelles after 7 d storage.

### Bio-safety of TGN/SHp/TPP-MLT micelles

Firstly, the cytotoxicity of TGN/SHp/TPP-MLT micelles was assessed by MTT assay. As shown in Fig. 3A and B, TGN/SHp/TPP-MLT micelles displayed minor cytotoxicity, and more than 90% bEnd.3 and PC-12 cells were alive at the highest concentration of 500 μM after incubation for 24 h.

**Fig. 3:** Bio-safety of TGN/SHp/TPP-MLT micelles. **A**, **B** Cell viability of bEnd.3 and PC-12 cells incubated with TGN/SHp/TPP-MLT micelles for 24 h. **C** Representative image of red blood cells incubated with water, saline and TGN/SHp/TPP-MLT micelles. **D** Hemolysis ratio of TGN/SHp/TPP-MLT micelles. **E** The influences of TGN/SHp/TPP-MLT micelles on bodyweight of Balb/c mice. **F** The influences of TGN/SHp/TPP-MLT micelles on the liver and kidney function of Balb/c mice (n = 6)

The hemolysis test was performed to assess the safety of TGN/SHp/TPP-MLT micelles for intravenous injection. As shown in Fig. 3C and D, the hemolysis ratios were generally low for several concentrations of TGN/SHp/TPP-MLT micelles, which were all lower than 1%, suggesting that TGN/SHp/TPP-MLT micelles would not cause damage to red blood cells.These results demonstrated a well hemocompatibility and TGN/SHp/TPP-MLT micelles could be further used for intravenous injection.

No significant change of body weight was observed in mice treated with TGN/SHp/TPP-MLT micelles in comparison to saline (Fig. 3E). The results of biochemical tests (Fig. 3F) showed that TGN/SHp/TPP-MLT micelles had good biological safety. The histopathological results (Fig. 3G) also showed that no abnormal changes in various organs occurred in mice treated with TGN/SHp/TPP-MLT micelles at TPP-MLT dose of 5 mg/kg.

### Cellular uptake

The prerequisites for TGN/SHp/TPP-MLT micelles to effectively ameliorate the injured neural cells during CIS are their specific distribution in brain tissues and then neural cells. The fluorescent probe cy3 was used to label blank TGN/SHp micelles, and TGN/SHp/cy3 micelles were prepared as TGN/SHp/TPP-MLT micelles. bEnd.3 cells are the immortalized mouse brain microvascular endothelial cells, highly expressing factor VIII and endothelial growth factor, etc. [34]. Therefore, bEnd.3 cells were used to construct in vitro BBB model. Firstly, the internalization of TGN/SHp/cy3 micelles was investigated. As shown in Fig. 4A, the fluorescent signals in cells treated with TGN/SHp/cy3 micelles and TGN/cy3 micelles were higher than those treated with micelles without TGN modification at each time point, including cy3 micelles and SHp/cy3 micelles. Additionally, the intracellular fluorescent intensity was measured by flow cytometry, and showed the similar results (Additional file 1: Fig. S4). TGN peptide modification increased the cellular uptake of micelles, whereas SHp peptide had no effects on internalization of micelles by bEnd.3 cells, as shown by low fluorescent signal in cells treated with SHp/cy3 micelles.

**Fig. 4:** Biodistribution of TGN/SHp/TPP-MLT micelles. **A** Representative fluorescence images of bEnd.3 cells incubated with TGN/SHp/cy3 micelles for for 0.5 and 2.0 h, TGN/cy3 micelles, SHp/cy3 micelles, cy3 micelles and free cy3 as control.Scale bar, 50 µm. **B** The transport ratios (%) of TGN/SHp/cy3 micelles across BBB model, TGN/cy3 micelles, SHp/cy3 micelles, cy3 micelles and free cy3 as control (n = 6, *P* > 0.05). **C** Representative fluorescence images of PC-12 cells incubated with TGN/SHp/cy3 micelles for for 0.5 and 2.0 h, TGN/cy3 micelles, SHp/cy3 micelles, cy3 micelles and free cy3 as control.Scale bar, 20 µm. **D** Representative fluorescent images of brain tissue in CIS mice treated with TGN/SHp/Dir micelles, Dir micelles as control. **E** The tissue distribution of TGN/SHp/TPP-MLT micelles in CIS mice at 0.5, 2.0 and 8.0 h after intravenous administration at a dose of 5 mg/kg TPP-MLT, free TPP-MLT and TPP-MLT micelles (n = 6, *P < 0.05). **F** TPP-MLT contents in ischemic and normal brain sides (n = 6, *P < 0.05)

Then, the ability of TGN/SHp/cy3 micelles across BBB was investigated. As shown in Fig. 4B, TGN/SHp/cy3 micelles across BBB model was time‐dependent and the transport percentages at 0.5, 1 and 2 h were 4.70 ± 0.96%, 7.54 ± 1.06% and 15.8 ± 2.12%, respectively. Similar transport percentage was also observed in TGN/cy3 micelles (*P* > 0.05). By contrast, the transport percentages were lower in micelles without TGN peptide modification, including SHp/cy3 micelles and cy3 micelles. SHp peptide modification had no effects on the transmembrane transport of micelles.

After across BBB, the specific distribution of TGN/SHp/cy3 micelles in neuronal cells undergoing apoptosis was investigated to confirm whether SHp stroke-homing peptide could increase drug accumulation in ischemia area. PC-12 cells were used to model the neuronal system [35]. As shown in Fig. 4C, the fluorescent signals in cells treated with TGN/SHp/cy3 micelles and SHp micelles were higher than those treated with micelles without SHp modification at each time point, including cy3 micelles and TGN/cy3 micelles. In addition, the fluorescent signals in cells treated with H_2_O_2_ + TGN/SHp/cy3 micelles were apparently higher than cells treated with PBS + TGN/SHp/cy3 micelles, confirming the stroke-homing effect of SHp peptide. The intracellular fluorescent intensity was measured by flow cytometry, and showed the similar results (Additional file 1: Fig. S6) that the increased intracellular fluorescent signals in oxidative stress-damaged cells treated with TGN/SHp/cy3 micelles and TGN/SHp/cy3 micelles. SHp peptide modification increased the cellular uptake of micelles by injuried neuronal cells, whereas TGN peptide had no effects on internalization of micelles, as shown by low fluorescent signals in cells treated with TGN/cy3 micelles.

### Bio-distribution of TGN/SHp/TPP-MLT micelles

TGN/SHp micelles were firstly observed by fluorescence imaging technique, and Dir was used to tap for micelles. 2 h after intravenous administration, the mice were sacrificed and brain tissues were dissected for ex vivo fluorescence imaging using the In-Vivo imaging system. As shown in Fig. 4D and Additional file 1: Fig. S7 (Semi-quantitative fluorescence intensity), compared with brain tissue isolated from CIS mice treated with Dir micelles, the stronger fluorescent signal was observed in brain tissue from CIS mice treated with TGN/SHp/Dir micelles, confirming its good distribution of TGN/SHp micelles in brain tissue of CIS experimental animal.

Then, the bio-distribution of TPP-MLT was investigated after injection at 0.5, 2 and 8 h. Heart, liver, spleen, lung, kidney and brain tissues were isolated, and TPP-MLT content was quantitatively determined by UPLC-MS/MS. As shown in Fig. 4E, litter TPP-MLT was detected in brain tissue of CIS mice treated with free TPP-MLT at a series of time points (0.5, 2 and 8 h). In contrast, the significantly increased TPP-MLT was detected in CIS mice treated with TGN/SHp/TPP-MLT micelles, which consistent the in vitro results of TGN/SHp/cy3 micelles across BBB at the help of TGN peptide. It should be noted that the increased TPP-MLT was detected in CIS mice treated with free TPP-MLT micelles, which was probably associated with the broken BBB [36]. The ability of TGN/SHp/TPP-MLT micelles to ischemic brain region was further investigated, and the results were shown in Fig. 4F. TPP-MLT contents in ischemic brain tissue were significantly higher than that in normal brain tissue of CIS mice treated with TGN/SHp/TPP-MLT micelles at a series of time points (0.5, 2 and 8 h). By contrast, no significantly increased TPP-MLT was detected in ischemic brain tissue compared with its distribution in normal brain tissue of MCAO mice treated with TPP-MLT micelles. This preferential distribution of TGN/SHp/TPP-MLT micelles in ischemic brain tissue was consistent the in vitro results of TGN/SHp/cy3 micelles specifically accumulated by the injuried PC-12 cells at the help of SHp peptide.

### Antioxidant and anti-apoptosis of TGN/SHp/TPP-MLT micelles

Compared with free MLT, TPP-MLT was more effectively to reduced intracellular ROS levels in H_2_O_2_-treated PC-12 cells. Antioxidant activity of TPP-MLT after encapsulated in TGN/SHp micelles was further investigated, free TPP-MLT as control. As shown in Fig. 5A, both free TPP-MLT and TGN/SHp/TPP-MLT micelles could reduce intracellular ROS levels in H_2_O_2_-treated PC-12 cells, and TGN/SHp/TPP-MLT micelles showed the better antioxidant activity. This result demonstrated that the increased TPP-MLT was internalized by H_2_O_2_-treated PC-12 cells after encapsulated in TGN/SHp micelles. After that, the JC-1 fluorescent probe was used to assess the changes of MMP in injuried PC-12 after treated with TGN/SHp/TPP-MLT micelles. As shown in Fig. 5B, the red/green fluorescent intensity ratio in H_2_O_2_-treated PC-12 cells was significantly enhanced after treated with free TPP-MLT and TGN/SHp/TPP-MLT micelles. Compared with free TPP-MLT, the larger enhancement of fluorescent intensity ratio was observed in H_2_O_2_-treated PC-12 cells treated with TGN/SHp/TPP-MLT micelles, further suggesting the increased TPP-MLT distribution contributed to relieving the oxidative stress in the mitochondria. Both MTT assay (Fig. 5C) and Calcein AM/Ethd-1 staining results (Fig. 5D and E) demonstrated that TGN/SHp/TPP-MLT micelles was more effective in improving the survival of H_2_O_2_-treated PC-12 cells compared with free TPP-MLT.

**Fig. 5:** In vivo efficacy of TGN/SHp/TPP-MLT micelles. **A** Expression levels of ROS in PC-12 cells treated with saline, TPP-MLT and TGN/SHp/TPP-MLT micelles. DCFH-DA fluorescent probes as ROS indicator. Scale bar, 50 μm. **B** The changes of mitochondrial membrane potential in PC-12 cells treated with saline, TPP-MLT and TGN/SHp/TPP-MLT micelles. Scale bar, 50 μm. **C** Cell viability of H_2_O_2_-stimulated PC-12 cells after treated with TGN/SHp/TPP-MLT micelles, free TPP-MLT as control (n = 6). **D** PC-12 cells were stained with calcein AM (green) and EthD-1 (red) to visualize live and dead cells. Scale bar, 200 μm. **E** Semi-quantitative fluorescent analysis of live and dead cells. **F** Flow cytometry-based apoptosis assay by the Annexin V-FITC Apoptosis Kit. PI, propidium iodide. **G** Western blot analysis of Cytochrome C in Mitochondria and Cytosol, Cleaved Caspase-3 and Cleaved Caspase-9 in H_2_O_2_-stimulated PC-12 cells treated with TGN/SHp/TPP-MLT micelles, free TPP-MLT as control. **H**–**K** Densitometric analysis of the western blot bands (n = 3, *P < 0.05)

Annexin V/PI staining was used to assess the effects of TGN/SHp/TPP-MLT micelles on H_2_O_2_-induced PC-12cell apoptosis. As shown in Fig. 5F, H2O2 treatment led to the increased apoptotic cells. TPP-MLT treatment effectively reduced apoptotic cells after cells being exposure to TPP-MLT for 24 h. By contrast, anti-apoptosis effect of TPP-MLT encapsulated in TGN/SHp/TPP-MLT micelles was further increased in PC-12 treated with H_2_O_2_, suggesting TGN/SHp micelles enhanced the drug transport into cells and then improved the therapeutical effect.

The effects of TGN/SHp/TPP-MLT micelles on mitochondria-mediated apoptotic protein expression were investigated, and the protein levels of Cytochrome C in mitochondria and cytosol, cleaved caspase-3 as well as cleaved caspase-9 were examined. As shown in Fig. 5G, I–K, the increased expression levels of cytosolic Cytochrome C, cleaved caspase-3 and cleaved caspase-9 were moderately inhibited in H_2_O_2_-treated PC-12 cells incubated with TGN/SHp/TPP-MLT micelles. In addition, the reduced expression of mitochondrial Cytochrome C was reversed by TGN/SHp/TPP-MLT micelles (Fig. 5G and H). By contrast, the effects of TPP-MLT on the protein expression of mitochondrial Cytochrome C, cytosolic Cytochrome C, cleaved caspase-3 and cleaved caspase-9 were less weak.

### In vivo pharmacodynamics

CIS injury could cause locomotor incoordination to the experimented mice. Neurological deficit score was adopted in this study to assess the behavioral changes in CIS mice treated with TGN/SHp/TPP-MLT micelles, free TPP-MLT as control. The mice treated with TGN/SHp/TPP-MLT micelles exhibited higher neurological scores in comparison to those treated with free TPP-MLT (Fig. 6A). The changes of ischemic region were also monitored with MRI in CIS mice treated with TGN/SHp/TPP-MLT micelles, free TPP-MLT as control. As shown in Fig. 6B, the red curve indicates the ischemic region. Compared with free TPP-MLT, the infarct area was remarkably reduced after TGN/SHp/TPP-MLT micelles treatment. The infarct volumes were further measured by TTC staining, which appeared redinteracting with dehydrogenase in normal tissues, and appeared pale in ischemic region due to the reduced dehydrogenase activity [31]. As shown in Fig. 6C, the normal brain tissue was uniformly red, while the ischemic brain tissue showed a pale infarct area. Compared with free TPP-MLT, TGN/SHp/TPP-MLT micelles were more effective to shrink infarct area and reduce infarct volume.

**Fig. 6:** In vivo efficacy of TGN/SHp/TPP-MLT micelles. **A** Neurological deficit scores of CIS mice treated with saline, TPP-MLT and TGN/SHp/TPP-MLT micelles. **B** T_2_-weighted images of ischemic brains in CIS mice treated with TPP-MLT and TGN/SHp/TPP-MLT micelles. The red curve indicates the infarct area. **C** TTC staining images of brain slices from CIS mice treated with TPP-MLT and TGN/SHp/TPP-MLT micelles. **D** and **E** Expression levels of SOD and MDA in infarct area of CIS mice treated with TPP-MLT and TGN/SHp/TPP-MLT micelles. **F** H&E staining sections of brain tissues of CIS mice treated with TPP-MLT and TGN/SHp/TPP-MLT micelles. Scale bar, 500 µm (n = 6, *P < 0.05)

SOD and MDA contents in brain tissues of CIS mice were measured after homogenization to evaluate the oxidative stress levels. As shown in Fig. 6D, compared with the sham operation (17.58 ± 0.52 U/mg prot), the SOD activity in the brain tissue of CIS mice were significantly reduced (15.35 ± 0.37 U/mg prot). After treatment, the significant increased SOD activity was observed in CIS mice treated with TGN/SHp/TPP-MLT micelles (TGN/SHp/TPP-MLT micelles *vs.* TPP-MLT, 15.86 ± 0.42 U/mg prot *vs.* 15.86 ± 0.42 U/mg prot). MDA level was significantly increased in the brain tissue of CIS mice (CIS *vs.* sham, 13.74 ± 1.98 nmol/mg prot *vs.* 3.24 ± 1.15 nmol/mg prot), suggesting that brain tissue lipid peroxidation increased after the occurrence of CIS. Compared with TPP-MLT treatment, TGN/SHp/TPP-MLT micelles effectively improved MDA level in the brain tissue of CIS mice (TGN/SHp/TPP-MLT micelles *vs.* TPP-MLT, 5.63 ± 2.31 nmol/mg prot *vs.*10.23 ± 2.34 nmol/mg prot) (Fig. 6E). H&E staining was used to analyze the pathological process of CIS. As shown in Fig. 6F, the brain tissues of the sham operation group have regular cell morphology, tight connections and normal structure; while the brain tissues of the CIS group showed disordered cell structure arrangement, increased gaps and edema-like appearance. Ischemic changes in cerebral cells were significantly reduced in the TPP-MLT and TGN/SHp/TPP-MLT micelles, with the TGN/SHp/TPP-MLT micelles having a more pronounced protective effect.

## Discussion

The BBB remains the primary challenge for brain-targeting drug delivery, and at the same time, the complexity of brain function and the sensitivity of neurons are easily to be affected by non-endogenous substances. After entering into the brain, drug is distributed throughout the brain tissue, which not only reduces the amount of drug reaching the lesion and weakens the therapeutic effect, but also potentially induce central system side effects. Therefore, the improved brain penetration and selective distribution within the brain is of great importance. The biodegradable nanoparticles mediated with appropriate targeting groups are promising candidates for CIS therapy due to their capability crossing the BBB and preferentially internalized by the oxidative stress-injured neurons.

Various dual-targeted drug delivery systems have been reported [37, 38], most of which were designed for tumor imaging and therapy. Chen et al. developed a nanoprobe simultaneously targeting to biotin receptor and carboxylesterase on HepG2 tumor [39]. Wang et al. developed nano-micelles imultaneously targeting to CD206 and CD44 receptor for the treatment of non-small cell lung cancer [40]. In these cases, both ligands target to the tumor cells, and two ligands can also play a cascade targeting effect [41]. Angiopep-2 peptide and EGFP-EGF1 protein modified on PEG-PCL nanoparticles help to penetrate BBB and then bind neuroglial cells [41]. In our this study, TGN peptide (TGNYKALHPHNG) was used to increase the BBB penetration of micelles, as Gao et al. reported [42]. After that, micelles were guided by SHp peptide (CLEVSRKNG) to oxidative stress-injured neural cells with up-regulated glutamate receptor during the occurrence of CIS [35].

Current strategies to achieve mitochondria-targeted drug delivery are based on the high potential to penetrate the mitochondrial membrane and its protein transport channels.Mitochondria have a bilayer membrane structure that separates the mitochondria into four parts with different properties and functions [43, 44]: (i) outer mitochondrial membrane, allowing free passage of molecules less than 5 kDa; (ii) the intermembrane space, which contains a variety of specific proteins; (iii) mitochondrial inner membrane with a lipid structure that is not easily permeable; and (iv) the mitochondrial lumen, which contains a variety of enzymes and coenzymes that regulate a variety of metabolic behaviors. The impermeable inner mitochondrial membrane can better maintain the ionic balance between the inner lumen and the cytoplasm. The mitochondria acquire the electrons they need through oxidation, then their own respiration causes the electrons to combine with oxygen to produce ATP, and the energy generated during oxidation is used for the transport of protons between the inside and outside of the mitochondria. The transport of protons inside and outside the membrane results in a transmembrane potential between 180 and 200 mV and a high pH value in the mitochondrial lumen. Compared to other organelles, mitochondria have a high transmembrane potential and exhibit high negative charges, which allows lipid-soluble cations to rapidly penetrate the mitochondrial bilayer membrane and enter and enrich in the mitochondria through charge interactions, such as triphenylphosphine (TPP), triphenylmethylphosphonium and tetraphenylphosphonium. TPP is a molecule composed of a single positively charged proton and three benzene rings, which are structurally stable and highly positively charged. It has been extensively used in mitochondrial targeting strategy, its three benzene rings forming delocalized positive charges and then penetrating the double hydrophobic membranes of mitochondria [43]. In our previous study, TPP was used to construct the stepwise-targeting chitosan oligosaccharide conjugate for acute kidney injury, and effectively ameliorate oxidative stress injury as well as improve renal function [20]. In this study, TPP was chemically grafted with the antioxidant MLT, resulting in the mitochondrial targeting properties of MLT, which was originally non-selective for organelles, and increasing the drug distribution in mitochondria. The quantitative test results were as expected, and the distribution of TPP-MLT in mitochondria was significantly higher than that of MLT.

## Conclusions

In conclusion, we have developed the cascade targeting TGN/SHp/TPP-MLT micelles for the treatment of CIS. Antioxidant MLT is delivered across the BBB, to the ischemic lesion site and ultimately to the intracellular mitochondria. It can scavenged the overproduced ROS to protect neuronal cells from oxidative stress injury during CIS occurrence. This strategy effectively ameliorates infarct volume and neurological deficit in MCAO induced cerebral ischemia–reperfusion injury. Its use provides new insights into the targeting treatment of CIS, and also provides potential applications for other inflammatory disorders.

## Supplementary Information

**Additional file 1.** Additional figures and table.
